# SOCS3 Gene Polymorphism and Hypertension Susceptibility in Chinese Population: A Two-Center Case-Control Study

This article has been retracted.

**DOI:** 10.1155/2021/8445461

**Published:** 2021-11-17

**Authors:** Dabin Kuang, Lichen Dong, Lingyun Liu, Meiling Zuo, Yuanlin Xie, Taoming Li, Zhousheng Yang

**Affiliations:** ^1^The Affiliated Changsha Hospital of Hunan Normal University, Changsha, Hunan 410006, China; ^2^Department of Pharmacy, The 921th Hospital of Joint Logistic Support Force of PLA, Hunan 410003, China; ^3^Department of Pharmacy, The People's Hospital of Guangxi Zhuang Autonomous Region, Guangxi Academy of Medicaid Sciences, Nanning 530021, China

## Abstract

Endothelial inflammation and vascular damage are essential risk factors contributing to hypertension. Suppressor of cytokine signaling 3 (SOCS3) is involved in the regulation of multiple inflammatory pathways. A large number of studies have shown that the anti-inflammatory effect of SOCS3 in hypertension, obesity, and allergic reactions has brought more insights into the inhibition of inflammation. Therefore, we selected a tagSNP of SOCS3 (rs8064821) to investigate whether they are contributing to the risk of hypertension in the Chinese population. In total, 532 patients with hypertension and 569 healthy controls were enrolled for two central of China. SOCS3 rs8064821 C>A polymorphism was genotyped using TaqMan assay. SOCS3 rs8064821 CA genotype was associated with an increased risk of hypertension (OR = 1.821, 95%CI = 1.276-2.600, *P* = 0.001). Rs8064821 A allele was associated with higher SOCS3 mRNA level in PBMCs from healthy donors. SOCS3 rs8064821 C>A polymorphism may contribute to the risk of hypertension in the Chinese population by regulating the expression of SOCS3.

## 1. Introduction

Hypertension is the leading contributing factor to all-cause global mortality Manosroi & Williams [1]. To date, hypertension affects over 1.2 billion individuals worldwide and has become the most critical and expensive public health problem Durham & Palmer [2]; Manosroi & Williams [1]; Rossier, Bochud, & Devuyst [3]; Samson, Ayinapudi, Le Jemtel, & Oparil [4]. It is the main risk factor for stroke (ischemic and hemorrhagic) and coronary artery disease Manosroi & Williams [1]; Rossier et al. [3]. In the past decades, considerable progress has been made in understanding that hypertension is not a disease but a syndrome. Studies have shown that most cases of hypertension are affected by environmental and disease factors, including drinking, smoking, changes in daily habits, hyperlipidemia, atherosclerosis, and diabetes. At the same time, genetic association studies have shown that genetic susceptibility has a great influence on the risk and prognosis of hypertension Kolifarhood et al. [5]. However, the genetic factors affecting hypertension are too complicated. Current research shows that it is a multigene-regulated disease. Identifying new risk sites for hypertension may help promote early diagnosis and therapeutic intervention of the disease.

Suppressor of cytokine signaling 3 (SOCS3) maps to chromosome 17q25.3 and consists of two exons Rancourt et al. [6]. SOCS3 is one of the suppressors of the cytokine signaling (SOCS) protein family. It modulates the outcome of infections and autoimmune diseases. And it has been shown to be involved in regulating signal transduction through a variety of cytokines, including insulin signaling and leptin signaling Carow & Rottenberg [7]. Recent studies have found that SOCS1 and SOCS3 are strong negative feedback regulators of cytokine signaling mediated by Janus kinase (JAK) signal transduction and transcription signal pathway activators and can play a key role in the development and progression of cancer and cardiovascular disease. The abnormal expression of SOCS3 in cancer cells, such as breast cancer Sun et al. [8], gastric cancer Zhou, Peng, & Xu [9], and small-cell lung cancer Zhao et al. [10], is related to the disorder of cell growth, migration, and death induced by a variety of cytokines and hormones in human cancers. It has been reported that inflammatory activation can upregulate SOCS3 expression and induce cardiovascular diseases Gan et al. [11]; Park et al. [12]; Wiejak, Dunlop, Mackay, & Yarwood [13]. However, some researches also confirmed that SOCS3 has a protective effect in limiting vascular inflammation. SOCS3 can reduce the ability of IL-6 signal transduction, thereby preventing vascular inflammatory diseases, such as atherosclerosis Ortiz-Munoz et al. [14]. And decreased SOCS3 leads to excessive production of inflammatory molecules in VSMC, which leads to enhanced vascular remodeling and vasoconstriction Tian et al. [15], while the mechanism of how SOCS3 affects hypertension remains unclear.

Obesity and chronic inflammation are key factors in the occurrence of hypertension, and they mutually cause and influence each other Mouton, Li, Hall, & Hall [16]. There is no report that the polymorphism of SOCS3 is associated with the risk of hypertension. Currently, Cid-Soto et al. found that the CAT haplotype in SOCS3 is associated with metabolic syndrome in Mestizos and correlated with protection against high blood pressure Cid-Soto et al. [17]. However, many studies have found that the polymorphisms of SOCS3 are related to obesity and serum lipid levels. Obesity is strongly associated with hypertension and cardiovascular disease Rahmouni, Correia, Haynes, & Mark [18]. Tessier et al. found that SOCS3 rs6501199, rs12944581, rs4969172, and rs4436839 polymorphisms affected the BMI of various ethnic groups Tessier, Fontaine-Bisson, Lefebvre, El-Sohemy, & Roy-Gagnon [19]. And another study has found that rs4969170 in SOCS3 was significantly associated with BMI positively Li et al. [20]. Previous studies have also found that rs4969168 Talbert et al. [21] and rs12953258 Yao et al. [22] polymorphisms are related to dyslipidemia in different populations.

However, whether the SOCS3 gene polymorphism is associated with the risk of hypertension has not been studied. The purpose of this study is to determine the predictive biomarkers of hypertension risk in the Chinese population and establish an experimental basis to improve the understanding of the causes and mechanisms of hypertension.

## 2. Materials and Methods

### 2.1. Study Participants

We recruited a total of 532 patients with hypertension and 569 healthy controls from 2 hospitals in 2 provinces of China. Among them, there are 274 hypertension patients and 285 control individuals included between January 2018 and December 2020 from the First People's Hospital of Jining City, Shandong Province. And there are 248 hypertension patients and 279 control individuals included between January 2020 and April 2021 from the People's Hospital of Guangxi Zhuang Autonomous Region. Eligible patients were men and women aged 18-80 years, with clinical evidence of hypertension as demonstrated by the World Health Organization that stipulates systolic blood pressure (SBP) ≥ 140 mmHg and/or diastolic blood pressure (DBP) ≥ 90 mmHg. Major exclusion criteria covered tumors or malignant diseases, severe hepatic or renal dysfunctions, and pregnancy. Control individuals with similar age and gender were selected from the physical examination center of the same hospital. The study protocols received approval from the People's Hospital of Guangxi Zhuang Autonomous Region. Informed consent was obtained from each participant or their guardian before the research.

### 2.2. Polymorphism Selection

Genetic polymorphisms were screened by the 1000 Genomes Project (http://www.internationalgenome.org/). Haploview 4.2 was used to select, and according to CHB and CHS, an unbalanced *R*^2^ value is more than 0.8, and the minimum allele frequency (MAF) was greater than 5%. F-SNP software (http://compbio.cs.queensu.ca/F-SNP/) was used to predict the possible functions of these selected sites. At last, we selected one site (rs8064821 C>A) of SOCS3 tagSNPs based on the above screening results and combined with the literature.

### 2.3. Genomic DNA Extraction and Genotyping

Genomic DNA was extracted from whole blood using the E.Z.N.A.™ Blood DNA Midi Kit (D3494, Omega) according to the standard protocol. DNAs were stored at −80°C until analysis. Genotype analysis was undertaken using TaqMan SNP Genotyping Assay from Applied Biosystems using 7500 Real-Time PCR System. And genotyping was performed utilizing TaqMan™ Genotyping Master Mix (4371355, Thermo) and TaqMan probes (C_43672951_10, Thermo) as recommended by the manufacturer.

### 2.4. Isolation of Peripheral Blood Mononuclear Cells (PBMCs)

30 healthy control subjects were recruited from the People's Hospital of Guangxi Zhuang Autonomous Region. An EDTA anticoagulant tube was used to obtain 5 mL of peripheral venous blood from each subject. The blood sample was diluted with an equal volume of phosphate-buffered saline (PBS). PBMCs were stratified using an equal volume of Histopaque-1077 (Sigma-Aldrich, St. Louis, MO) and separated by centrifugation (400 × g) for 30 minutes at room temperature.

### 2.5. RNA Isolation and Real-Time PCR

RNAiso Plus reagents (9109, TAKARA) were utilized to extract the total RNA from PBMCs. The absorbance of the extracted RNA was measured on a spectrophotometer. Subsequently, the RNA samples were converted to cDNA using PrimeScript RT Reagent Kit (RR036A, TAKARA) according to the manufacturer's instruction. The mRNA levels of SOCS3 in the samples were quantified with ABI 7500 Real-Time PCR System using SYBR Premix EX Taq System (RR820A, TAKARA) following the manufacturer's instruction. The primer sequences involved in the experiment were as follows: SOCS3, forward, 5′-CACATGGCACAAGCACAAGA-3′; reverse, 5′-AAGTGTCCCCTGTTTGGAGG-3′; GAPDH, forward, 5′-CTGCACCACCAACTGCTTAG-3′, reverse, 5′-AGGTCCACCACTGACACGTT-3′. The expression of target genes was analyzed using the 2^-*ΔΔ*Ct^ method.

### 2.6. Statistical Assay

All data are expressed as mean ± SD. SPSS 19.0 (version 19.0 for Windows; Chicago, IL, USA) was used for statistical analysis. Hardy–Weinberg equilibrium was compared by the *χ*^2^ test. Unpaired two-tailed Student's *t*-test was used to determine statistical significance between two groups' normally distributed continuous variables. And for multiple group comparison, one-way ANOVA analysis was used. Logistic regression method was used to analyze the effect of SOCS3 polymorphism on the risk of hypertension adjusting for multiple cardiovascular risk factors. ORs and 95% CIs calculated from the logistic regression analysis were used to assess the strength of association between SOCS3 polymorphisms and hypertension risk. A two-sided *P* value < 0.05 was considered statistically significant.

## 3. Results

### 3.1. Population Characteristics

The basic clinical characteristics of the 532 hypertension patients and 569 healthy controls are shown in Table 1. Patients with hypertension showed significantly higher BMI, SBP, DBP, fasting blood glucose (FBG), total cholesterol (TC), high-density lipoprotein cholesterol (HDL-C), and low-density lipoprotein cholesterol (LDL-C) compared to the controls. Hypertension patients also showed a higher prevalence of smoking. No significant differences in gender and age were observed between patients and controls (*P* > 0.05).

### 3.2. Association of SOCS3 rs8064821 C>A Polymorphisms and Risk for Hypertension in the South of China

Genotype distribution of the SOCS3 rs8064821 polymorphisms in both controls and hypertension patients was in agreement with the Hardy-Weinberg equilibrium (HWE) (control: HWE = 0.347, and hypertension: HWE = 0.812).  Table 2 shows the association between SOCS3 polymorphisms and hypertension risk in the south of China. Logistic regression analysis showed that the rs8064821 TT genotypes were associated with increased risk of hypertension (additive model: AA: odds ratio (OR) = 2.558, 95%confidence interval (CI) = 1.150-5.690, *P* = 0.021; dominant model: OR = 1.509, 95%CI = 1.067-2.133, *P* = 0.020; and recessive model: OR = 2.232, 95%CI = 1.017-4.897, *P* = 0.045). And after adjustment for age, gender, BMI, smoking history, FBG, and dyslipidemia, the result was also significant (additive model: CA: odds ratio (OR) = 2.647, 95%confidence interval (CI) = 1.391-5.038, *P* = 0.003; AA: odds ratio (OR) = 5.776, 95%confidence interval (CI) = 1.613-20.682, *P* = 0.007; dominant model: OR = 2.943, 95%CI = 1.584-5.466, *P* = 0.001; and recessive model: OR = 3.729, 95%CI = 1.119-12.426, *P* = 0.032).

### 3.3. Association of SOCS3 rs8064821 C>A Polymorphisms and Risk for Hypertension in the North of China

Similar to the south of China, genotype distribution of the SNP was in accordance with HWE in the controls and patients (control: HWE = 0.607, and hypertension: HWE = 0.654, respectively). Logistic regression analyses revealed that hypertension risk was increased significantly in the CA genotype of rs8064821 polymorphism than the CC genotype (additive model: CA: OR = 1.565, 95%CI = 1.100-2.228, *P* = 0.013; dominant model: OR = 1.592, 95%CI = 1.135-2.232, *P* = 0.007) as shown in Table 3. And after adjustment, the association was still significant (additive model: CA: OR = 1.965, 95%CI = 1.210-3.191, *P* = 0.006; dominant model: OR = 1.854, 95%CI = 1.166-2.947, *P* = 0.009).

### 3.4. Association of SOCS3 rs8064821 C>A Polymorphisms and Risk for Hypertension in Combined Subjects

Then, we aggregated and analyzed all the data from the two centers in Guangxi and Shandong Province. We found that the polymorphism of rs8064821 was associated with the risk of hypertension. Logistic regression analysis showed that the rs8064821 CA and AA genotypes were associated with increased risk of hypertension (additive model: CA: OR = 1.479, 95%CI = 1.150-1.902, *P* = 0.002; AA: OR = 2.110, 95%CI = 1.225-3.634, *P* = 0.007; dominant model: OR = 1.548, 95%CI = 1.215-1.971, *P* < 0.001; and recessive model: OR = 1.811, 95%CI = 1.061-3.091, *P* = 0.029, Table 4). However, no significant association was observed after adjustment for the recessive model, while the associations for additive and dominant models were still significant (additive model: CA: OR = 1.821, 95%CI = 1.276-2.600, *P* = 0.001; AA: OR = 2.143, 95%CI = 1.042-4.410, *P* = 0.038; dominant model: OR = 1.836, 95%CI = 1.326-2.619, *P* < 0.001).

### 3.5. Association of SOCS3 rs8064821 C>A Polymorphism with SOCS3 Expression

In order to explore whether the genetic polymorphism of rs8064821 is associated with the mRNA expression level of SOCS3, we analyzed the relevant information in the Genotype-Tissue Expression (GTEx) database. As shown in Figure 1, rs8064821 A allele was associated with increased SOCS3 mRNA in adipose tissue, such as adipose subcutaneous and adipose visceral (the relative expression median: CC: -0.09489, CA: 0.2325, AA: 0.4881, *P* = 2.21*e* − 8; CC: -0.07741, CA: 0.2782, AA: -0.02204, *P* = 4.99*e* − 8, respectively). Similarly, in artery tissues, the mRNA expression level of SOCS3 has the same correlation with the rs8064821 genotype (artery aorta: CC: -0.08084, CA: 0.4946, AA: 0.05818, *P* = 1.33*e* − 5; artery coronary: CC: -0.08208, CA: 0.2727, AA: 0.6382, *P* = 1.02*e* − 2; and artery tibial: CC: -0.1052, CA: 0.2445, AA: 0.2314, *P* = 1.54*e* − 7, respectively). And in whole blood, the relative expression level of SOCS3 was higher in the CA and AA genotypes than in the AA genotype (CC: -0.1179, CA: 0.2184, AA: 0.3954, *P* = 4.1*e* − 8).

To further verify the analysis results of the database, we determined the mRNA expression level of SOCS3 in 30 randomly selected healthy controls. PBMCs from 21 subjects carrying the rs8064821 CC genotype were collected, the others (*n* = 9) bearing the rs8064821 CA genotype. No PBMCs from individuals with the rs8064821 AA genotype were collected. As compared with PBMCs carrying the rs8064821 CC genotype, the CA genotype showed significantly higher levels of SOCS3 mRNA expression (*P* < 0.05, Figure 2).

## 4. Discussion

In this study, we investigated whether SOCS3 gene polymorphism was involved in the risk of hypertension in the Chinese population using individuals from two centers. The results presented here represent that rs8064821 C>A polymorphism contributed to the risk of hypertension. Our results demonstrated that the rs8064821 CA genotype was associated with an increased risk of hypertension in the Chinese Han population. Moreover, we observed that the rs8064821 C>A polymorphism affected the expression level of SOCS3 in healthy subjects, with subjects heterozygote for the rs8064821 genotype showing significantly higher mRNA level of SOCS3 than the AA genotype in PBMCs.

SOCS protein is usually expressed at low levels under basal conditions, but it is rapidly induced by inflammatory factors. Induced SOCS3 can block IL-6/JAK/STAT activity, forming a classic negative feedback loop Moshapa, Riches-Suman, & Palmer [23]. SOCS3 inhibits the activation of JAK/STAT induced by IL-6 by directly inhibiting JAK kinase activity, thereby preventing the binding of the substrate and ATP Kershaw et al. [24]. Durham and Palmer found that IL-6 activates JAK-STAT signaling to induce the transcription of proinflammatory and proantigen genes, and SOCS3 restricts IL-6 signaling, which resists the progression of pulmonary arterial hypertension (PAH) Durham & Palmer [25]. Damage to endothelial function and vascular inflammation are key factors in the onset of hypertension. Recently, a study also found that SOCS3 expression induced by angiotensin II regulates the effect of inflammation. Knockout of SOCS3 expression in bone marrow-derived cells can prevent systemic angiotensin II-induced vascular dysfunction and then affect the angiotensin II involved in the control of blood pressure and cardiac contractility Li, Kinzenbaw, Modrick, Pewe, & Faraci [26]. SOCS3 plays an important role in maintaining the vascular function, and the correlation between the polymorphism of SOCS3 and cardiovascular disease has also been partially studied. A recent study found a significant association between SOCS3 rs7221341 and decreased risk of high blood pressure. And the SOCS3 rs7221341, rs4669168, and rs9914220 polymorphisms were associated with type 2 diabetes and high waist circumference in Mexican Amerindians Cid-Soto et al. [17]. In this study, we found that the SOCS3 rs8064821 C>A polymorphism is associated with the risk of hypertension. The risk of hypertension of the CA genotype is significantly higher than that of the CC genotype.

Some previous studies have found that the polymorphism of SOCS3 rs8064821 is related to some diseases, such as cancer and obesity. Reid-Lombardo et al. found that in patients with resection of pancreatic cancer, the SOCS3 rs8064821 C>A polymorphism was associated with a survival advantage of approximately 10 months compared with noncarriers Reid-Lombardo et al. [27], while Jiang et al. analyzed the association between the genetic polymorphism of the SOCS3 gene and the incidence and progression of hepatocellular carcinoma (HCC) Jiang et al. [28]. They confirmed that the genotype frequencies of rs12953258 and rs8064821 were not significantly different between HCC and the control group. However, for the rs4969170 polymorphism, the prevalence of GG in HCC patients was higher than that in the control group. Boyraz et al. found that SOCS3 rs8064821 G>T polymorphism is associated with obesity parameters in children. Their results showed that the GG genotype frequency at rs8064821 locus is significantly higher in the nonmetabolic syndrome obese group than in the metabolic syndrome obese group Boyraz et al. [29]. In another study, the authors did not find the correlation between rs4969169, rs12953258, and rs8064821 and general obesity and central obesity in normal female twins and also not related to the two indexes of insulin sensitivity Jamshidi et al. [30]. In this study, we found that the SOCS3 rs8064821 C>A polymorphism is associated with the risk of hypertension in the populations of the two centers. Meanwhile, the analysis after summarizing all subjects also yielded similar results. The risk of hypertension of the CA or AA genotype is about 1.8-fold than that of the CC type.

Hypertension is a disease affected by multiple factors, and the activation of inflammatory pathways plays an important role in its pathogenesis. SOCS3 modulates the inflammatory pathways responsible for vascular stability. Recently, Zhang et al. analyzed the data of blood transcriptomics in the GEO database and collected clinical subjects for verification. They found that compared with healthy controls, patients with stable coronary artery disease (CAD) and acute coronary syndrome (ACS) had significantly lower levels of SOCS3 expression. And the probe expression levels of SOCS3 were significantly upregulated in patients with ST-segment elevation myocardial infarction (STEMI) when compared to stable CAD patients Zhang et al. [31]. Ali et al. used ELISA to detect SOCS3 levels in serum. Their results showed higher SOCS3 levels in the hypertensive group versus normotensive Ali, Ali, Farhat, & Fatima [32]. A recent study found that SOCO3 has a certain value in predicting the efficacy of pregnancy-induced hypertension by analyzing the plasma SOCS3 levels before and after being treated with nifedipine in patients with pregnancy-induced hypertension Zhao, Ai, Wu, & Dong [33]. These researches suggest that the expression level of SOCS3 may be related to the pathological process of hypertension. By analyzing the data in the GTEx database, we found that the expression level of the rs8064821 CA and AA genotype SOCS3 in adipose tissue, artery, and whole blood was significantly higher than that of the CC genotype. What is more, we found a significant upregulation of SOCS3 in the CA genotype than in the CC genotype in PBMCs. Previously, we used the F-SNP online tool to predict the function of the polymorphism of rs8064821. It was found that this site may affect the binding of transcription factors, which in turn affects the expression of SOCS3. Based on the results of this experiment, we speculate that the SOCS3 rs8064821 C>A polymorphism may affect the risk of hypertension by affecting the expression level of SOCS3.

While our results are promising, the intensity of current research is accompanied by some limitations. We would like to enlist all the limitations of the study:

1. Although this is a two-center study, the participants in this study are restricted to the Guangxi and Shandong populations in China. Therefore, the current research results cannot be generalized to other racial/ethnic groups. Due to the small sample size, although the calculation meets the statistical power, there may still be deviations. Therefore, large-scale, high-quality research should be conducted in the future to verify these findings
2. Due to the low frequency of the rs8064821 AA genotype (about 4% in healthy people), we did not collect samples of the AA genotype when studying the SOCS3 mRNA expression levels of different genotypes. We did not measure the expression levels of SOCS3 mRNA in peripheral blood PBMC cells of people with the AA genotype, thus preventing us from exploring the impact of the AA genotype on human phenotypes. These data may lead to different conclusions about the relationship between SOCS3 rs8064821 and its mRNA expression. Further research needs to expand the RNA sample to verify our conclusions
3. The conclusion drawn here lacks universality. In our study, the polymorphism of rs8064821 may affect the mRNA expression of SOCS3, but the mechanism is unclear. Although the previous studies have confirmed that the high expression of SOCS3 is relevant to the increase of inflammatory factors and blood lipid levels, whether the polymorphism of rs8064821 is related to it needs further experiments to verify. Therefore, we need in vivo and in vitro studies to confirm the mechanism of the association between rs8064821 and the risk of hypertension

## 5. Conclusion

In conclusion, here, we provide the possibility of the SOCS3 rs8064821 C>A polymorphism in predicting hypertension risk. Well-designed case-control studies with large samples are needed to confirm these findings. Our study serves as a basis for future replication studies in independent populations or functional studies of SOCS3 in hypertension risk.

## Figures and Tables

**Figure 1:** Effect of SOCS3 rs8064821 C>A polymorphism on SOCS3 mRNA expression in tissues from healthy normal donors.

**Figure 2:** Effect of the SOCS3 rs8064821 C>A polymorphism on SOCS3 mRNA expression in PBMCs.

**Table 1:** General characteristics of the hypertension patients and controls.

Characteristics	Guangxi Province			Shandong Province			Combined subjects		
	Control	Hypertension	*P*	Control	Hypertension	*P*	Control	Hypertension	*P*
Gender	279	248		290	274		569	522	
Male (%)	168 (60.2%)	152 (61.3%)		159 (54.8%)	135 (49.3%)		327 (57.5%)	287 (55.0%)	
Female (%)	111 (39.8%)	96 (38.7%)	0.801	131 (45.2%)	139 (50.7%)	0.187	242 (42.5%)	235 (45.0%)	0.408
Age (years)	53 ± 8	53 ± 8	0.231	53 ± 7	53 ± 8	0.394	53 ± 8	53 ± 8	0.146
BMI (kg/m^2^)	22.67 ± 1.52	25.27 ± 2.77	<0.001	23.40 ± 2.70	24.81 ± 3.61	<0.001	23.04 ± 2.23	25.02 ± 3.24	<0.001
SBP (mmHg)	121 ± 12	136 ± 20	<0.001	121 ± 11	139 ± 18	<0.001	121 ± 11	138 ± 19	<0.001
DBP (mmHg)	75 ± 7	84 ± 12	<0.001	76 ± 8	81 ± 13	<0.001	76 ± 8	82 ± 13	<0.001
Smoking history (%)	34 (12.2%)	61 (24.6%)	<0.001	46 (15.9%)	77 (28.1%)	<0.001	83 (14.6%)	138 (26.4%)	<0.001
FBG (mmol/L)	4.58 ± 0.47	5.5 ± 1.19	<0.001	4.91 ± 0.65	5.44 ± 0.83	<0.001	4.75 ± 0.59	5.46 ± 1.01	<0.001
TG (mmol/L)	1.18 ± 0.40	2.04 ± 1.32	<0.001	1.33 ± 0.79	1.45 ± 0.95	0.127	1.26 ± 0.64	1.73 ± 1.18	<0.001
TC (mmol/L)	4.56 ± 0.61	5.00 ± 0.94	<0.001	4.21 ± 1.11	4.70 ± 1.10	<0.001	4.38 ± 0.92	4.85 ± 1.04	<0.001
HDL-C (mmol/L)	1.24 ± 0.35	1.24 ± 0.51	1	1.23 ± 0.32	1.42 ± 0.57	<0.001	1.24 ± 0.33	1.33 ± 0.55	<0.001
LDL-C (mmol/L)	2.55 ± 0.64	3.07 ± 1.64	<0.001	2.17 ± 0.86	2.40 ± 0.76	0.001	2.36 ± 0.78	2.72 ± 1.30	<0.001

BMI: body mass index; SBP: systolic blood pressure; DBP: diastolic blood pressure; FBG: fasting blood glucose; TC: total cholesterol; TG: triglyceride; HDL-C: high-density lipoprotein cholesterol; LDL-C: low-density lipoprotein cholesterol.

**Table 2:** Association between SOCS3 rs8064821 C>A polymorphism and hypertension risk in Guangxi Province.

Models	Genotypes	Control, *n* = 279 (%)	Hypertension, *n* = 248 (%)	Unadjusted OR (95% CI)	*P* value	Adjusted OR^∗^ (95% CI)	Adjusted *P* value^∗^
rs8064821 C>A		HWE = 0.374	HWE = 0.812				
Additive	CC	171 (61.3)	127 (51.2)	1.00 (reference)		1.00 (reference)	
	CA	98 (35.1)	102 (41.1)	1.401 (0.978-2.009)	0.066	2.647 (1.391-5.038)	0.003
	AA	10 (3.6)	19 (7.7)	2.558 (1.150-5.690)	0.021	5.776 (1.613-20.682)	0.007
Dominant	CC	171 (61.3)	127 (51.2)	1.00 (reference)		1.00 (reference)	
	CA/AA	108 (38.7)	121 (48.8)	1.509 (1.067-2.133)	0.020	2.943 (1.584-5.466)	0.001
Recessive	CC/CA	269 (96.4)	229 (92.3)	1.00 (reference)		1.00 (reference)	
	AA	10 (3.6)	19 (7.7)	2.232 (1.017-4.897)	0.045	3.729 (1.119-12.426)	0.032

OR: odds ratio; CI: confidence interval. ^∗^Adjusted for age, gender, BMI, smoking history, FBG, and dyslipidemia.

**Table 3:** Association between S0CS3 rs8064821 C>A polymorphism and hypertension risk in Shandong Province.

Models	Genotypes	Control, *n* = 290 (%)	Hypertension, *n* = 274 (%)	Unadjusted OR (95% CI)	*P* value	Adjusted OR^∗^ (95% CI)	Adjusted *P* value^∗^
rs8064821 C>A		HWE = 0.607	HWE = 0.654				
Additive	CC	187 (64.5)	146 (53.3)	1.00 (reference)		1.00 (reference)	
	CA	90 (31.0)	110 (40.1)	1.565 (1.100-2.228)	0.013	1.965 (1.210-3.191)	0.006
	AA	13 (4.5)	18 (6.6)	1.773 (0.841-3.738)	0.132	1.264 (0.456-3.502)	0.653
Dominant	CC	187 (64.5)	100 (38.0)	1.00 (reference)		1.00 (reference)	
	CA/AA	103 (35.5)	163 (62.0)	1.592 (1.135-2.232)	0.007	1.854 (1.166-2.947)	0.009
Recessive	CC/CA	277 (95.5)	256 (93.4)	1.00 (reference)		1.00 (reference)	
	AA	13 (4.5)	18 (6.6)	1.498 (0.720-3.119)	0.280	0.979 (0.361-2.659)	0.967

OR: odds ratio; CI: confidence interval. ^∗^Adjusted for age, gender, BMI, smoking history, FBG, and dyslipidemia.

**Table 4:** Association between SOCS3 rs8064821 C>A polymorphism and hypertension risk in combined subjects.

Models	Genotypes	Control, *n* = 569 (%)	Hypertension, *n* = 522 (%)	Unadjusted OR (95% CI)	*P* value	Adjusted OR^∗^ (95% CI)	Adjusted *P* value^∗^
rs8064821 C>A		HWE = 0.786	HWE = 0.368				
Additive	CC	358 (62.9)	273 (52.3)	1.00 (reference)		1.00 (reference)	
	CA	188 (33.0)	212 (40.6)	1.479 (1.150-1.902)	0.002	1.821 (1.276-2.600)	0.001
	AA	23 (4.1)	37 (7.1)	2.110 (1.225-3.634)	0.007	2.143 (1.042-4.410)	0.038
Dominant	CC	358 (62.9)	273 (52.3)	1.00 (reference)		1.00 (reference)	
	CA/AA	211 (37.1)	249 (47.7)	1.548 (1.215-1.971)	<0.001	1.863 (1.326-2.619)	<0.001
Recessive	CC/CA	546 (95.9)	485 (92.9)	1.00 (reference)		1.00 (reference)	
	AA	23 (4.1)	37 (7.1)	1.811 (1.061-3.091)	0.029	1.696 (0.839-3.428)	0.141

OR: odds ratio; CI: confidence interval. ^∗^Adjusted for age, gender, BMI, smoking history, FBG, and dyslipidemia.

## Data Availability

he research data used to support the findings of this study are available from the corresponding author upon request.
